The article "Deep Learning-Based Music Quality Analysis Model" was retracted in 2023. Reasons: signs of a paper mill; suspected computer-generated content; unreliable results or conclusions; lack of ethics approval or compliance.

# Deep Learning-Based Music Quality Analysis Model

**DOI:** 10.1155/2022/6213115

**Published:** 2022-06-13

**Authors:** Jing Jing

**Affiliations:** Music Teaching Department, Zhengzhou Preschool Education College, Zhengzhou 450000, China

## Abstract

In order to build an efficient and effective deep much quality recognition model, a decision fusion method by leveraging the advantages of shallow learning and deep learning is formulated. In the literature, shallow learning is a traditional music-related quality recognition method, that is, artificial statistical feature extraction and recognition are designed. Meanwhile, our deep learning module leverages the so-called PCANET network to implement the feature extraction process, and subsequently takes the spectrogram describing the music-related information as the network input. First, a variety of task classifications for the music signal problem are divided. Afterward, the optimization and adoption of deep learning in the two major problems of music feature extraction and sequence modeling are introduced. Finally, a music application is presented to illustrate the practical application of deep learning in music quality evaluation. The shallow learning features and deep learning features are seamlessly combined into the SVM model for music quality modeling, based on which differential voting mechanisms are leveraged to realize the fusion of decision-making layers. Extensive experimental results have shown that the music quality recognition rate by this method can be significantly improved on our own compiled library and the Berlin database. Besides, it exhibits obvious advantages compared with the competitors.

## 1. Introduction

Music quality analysis is a research hotspot in the field of pattern recognition. It has become an indispensable technology for the development of new human-computer interaction systems and artificial intelligence [1]. Music quality evaluation technology can be mainly divided into three stages: speech signal collection, feature extraction, and quality score calculation [2], among which the key modules are feature extraction and quality score calculation. Researchers have carried out detailed analysis and research on acoustic feature extraction for the past decades. Acoustic features mainly include prosodic features, frequency domain features, and sound quality features [3]. These features play a key role in traditional music quality recognition, combined with other features. The feature selection algorithm can achieve excellent music quality recognition performance for multiple datasets. It is worth mentioning that researchers have attempted to combine the acoustic features of the temporal and frequency domains. They have proposed a spectrogram feature extraction method, which was applied to speech recognition [4] and speech emotion recognition related fields [5].

The article "Deep Learning-Based Music Quality Analysis Model" was retracted in 2023. Reasons: signs of a paper mill; suspected computer-generated content; unreliable results or conclusions; lack of ethics approval or compliance.

In terms of recognition models, it is from shallow learning support vector machine (SVM) [6], hidden Markov model (HMM) [7], and Gaussian mixture model (GMM) [8] to deep learning convolutional neural network (CNN) [9], deep belief network (DBN) [10], and recurrent neural network (RNN) [11]. Compared with traditional machine learning models, deep learning can extract high-level features. It has achieved excellent performance in the field of computer vision and speech recognition in recent years. Among them, convolutional neural networks have achieved unprecedented success in music quality recognition, image recognition, and other domains [10]. Many researchers have also introduced deep learning into SER tasks. Zhu et al. [10] leveraged the deep belief network to automatically extract the speech emotion features, combined with the speech emotion features of continuous multiple frames to construct a high-dimensional feature. They are finally input into the support vector machine (SVM) for classification. Hong et al. [12] extracted salient features based on the well-known CNN network, which can substantially improve the performance of SER emotion recognition in various complex sceneries. Experiments have shown that this method has high robustness and stability. Liao et al. [13] trained an improved CNN model, which can extract significant speech emotion features, thereby improving the emotion recognition rate. Wang et al. [14] extracted high-level features and applied RNN for music quality prediction. It can achieve a recognition accuracy of 62% on the IEMOCAP database. Yao et al. [15] proposed a data preprocessing algorithm to acquire more data by changing the size of the spectrogram and input it into the deep neural network model AlexNet. It obtained an average accuracy of 48.8% on the IEMOCAP dataset. [16] investigated the feedforward neural networks and recurrent neural networks and their variants suitable for SER tasks. This technique verified the effectiveness of deep learning structures in paralinguistic speech recognition. [17] proposed a speech-based music quality recognition method using convolutional neural network to identify spectrogram features. More specifically, the grayscale spectrogram features were extracted, and subsequently, the Gabor wavelet and block PCA were leveraged for feature extraction and dimension reduction. It is fed into CNNs for music quality recognition and classification, wherein impressive results have been achieved. Although deep learning has achieved satisfactory results on SER, the traditional speech emotion recognition (shallow learning) in the past is still valuable. The shallow learning model exhibits fast training speed and few parameters, based on which the extracted features are targeted. The deep learning network has a complex structure, requires a large amount of training data, and is complicated and expensive to adjust parameters. Pointed out that deep learning does not require manual parameter tuning and lacks the guidance of prior knowledge. It proposes a method of leveraging shallow learning to guide deep learning, which indicates that shallow learning still has an unprecedented significance. For the speech emotion recognition problem, although it is the era of big data, the effective data obtained is limited, and shallow learning has advantages in small-sample datasets. Complementary advantages are a topic worthy of study.

The article "Deep Learning-Based Music Quality Analysis Model" was retracted in 2023. Reasons: signs of a paper mill; suspected computer-generated content; unreliable results or conclusions; lack of ethics approval or compliance.

Herein, we in this paper propose a speech emotion recognition model that integrates deep learning and shallow learning. Our method is suitable for small-sample speech. Two recognition models are constructed: traditional speech recognition—shallow learning and deep learning framework—PCANET model. Our method finally proposes the two models to fuse to form an effective decision-making layer. Our proposed research goal is to make full use of the advantages of shallow learning and deep learning to avoid deficiencies and improve the music quality recognition rate and robustness. Traditional auditory features are targeted but highly objective. Deep letters mesh can automatically extract characteristic, but they will be inclined by the number of match and parameters. Through an effective settlement liquefaction method, the gain of both can be exhaustively utilized to obtain a steady and lofty rondo quality notice valuation. An overview of our discourse ignorant and profound fashion union framework is presented in Figure 1.

## 2. Related Work

### 2.1. Acoustic Feature Extraction

Music is used to transfer messages, intentions, and emotions, and is the most familiar way for humans to convey messages. Music has the characteristics of large, precise, and accurate information contained. With the development of multimedia information processing technology and the enhancement of computer data processing capability, audio processing technology has received attention and has been widely applied in many domains. The practical applications of speech recognition, speech synthesis, and speaker recognition are constantly and widely entering life. Meanwhile, music-related technology has become an important part of artificial intelligence and one of the main directions of multimedia application. Music signals have a larger range than speech signals, and there are many important and interesting research directions, such as audio scene analysis. In the past few decades, MFCC has been widely applied in audio analysis tasks, and its extraction steps are standardized. However, the disadvantage of this approach is that the artificially constructed features may not be optimal for the target task. The essence of filtering the sound signal is to incorporate different weights to it, and these weights can be learned by the neural network without artificial design. The deep neural network has the ability to automatically extract features. In this way, the above two separation problems can be jointly optimized. Furthermore, through the deep learning method, the steps of FFT transformation and Mel filtering can be discarded. Also, the neural network can directly perform feature learning on the sound sequence, completely abandoning all previous feature engineering operations. In feature extraction, after introducing the deep learning method, on the one hand, the neural network of the frequency domain filter bank can be constructed on the Mel filter bank. If shape constraints are introduced, filter gain, center frequency, and bandwidth are three learnable parameters. For triangular window filters, sigmoid curves and straight lines can be leveraged to fit triangular windows to ensure global differentiability, Gaussian window filter or filter without shape constraint. On the spectral reconstruction task, the unconstrained filter bank performs better, while on the audio scene classification task, the shape-constrained filter bank performs better. Further analysis of the learned filters demonstrates that the learnable filter banks tend to integrate more low-frequency information. Another aspect is to improve an end-to-end audio feature extraction method. For example, the well-known TCNN is proposed that integrates a temporal signal processing unit. It can use temporal convolution + temporal pooling + nonlinear transformation. WaveNet proposes that layer-by-layer neighborhood convolution and temporal pooling nonlinear transformation can be leveraged. It should be observable that the DCT transformation in the conventional method will lose the structural information of different music, so it does not perform well in the deep model. The most widely used features are the log-mel spectrum and the constant-Q spectrum. And the latter one is commonly used in music information retrieval tasks.

The article "Deep Learning-Based Music Quality Analysis Model" was retracted in 2023. Reasons: signs of a paper mill; suspected computer-generated content; unreliable results or conclusions; lack of ethics approval or compliance.

### 2.2. Deep Learning

Deep learning is a deep machine learning architecture whose depth is indicated in multiple transformations of features. The commonly used deep model is a multilayer neural network. Each layer of the neural network will input some nonlinear mapping. Through the stacking of multiple layers of nonlinear mapping, very abstract features can be calculated in the deep neural network to conduct classification. For example, in the convolutional neural network used for image analysis, the pixel value of the original image is directly inputted. Meanwhile, the first layer of neural network can be regarded as an edge detector, and the second layer of neural network can detect the combination of edges. It can obtain multiple basic modules; the networks after the third layer will combine these basic modules and finally detect the target to be identified. The deep learning makes there is no need to select and transform the features separately in many applications. We just have to input the original data into the model, and the model will give the feature representation suitable for classification through learning. The re-emergence of neural networks began in 2006. Hinton et al. proposed the training algorithms of deep belief network (DBN) and restricted Boltzmann machine (RBM). He applied the DBN to handwritten characters recognition, and highly competitive results can be observed. The authors proposed an unsupervised learning method that can be leveraged to initialize the parameters layer by layer, and subsequently the supervised learning method is leveraged to fine-tune the training method of the entire network. This scheme can effectively solve the problem of deep neural network learning. Such a training method can initialize the neural network using an optimal initial value, and it is convenient to converge to a better local extremum. In the following years, deep neural networks became popular and were generalized as “deep learning.” Many deep learning training algorithms were proposed, such as parameter initialization methods, new activation functions, and dropout (discard) training methods. These techniques can better solve the problems of overfitting and difficult training of traditional neural networks when the deep architecture is complicated. Meanwhile, the development of computers and the Internet has also made it feasible to accumulate unprecedented amounts of data to train neural networks in computer vision tasks such as image recognition. In the ImageNet competition in 2012, Krizhevsky et al. proposed the convolutional neural networks to increase the accuracy rate by 10%, which for the first time significantly surpassed the learning mode of hand-designed features with shallow model. It also introduces deep learning techniques in the industry. In 2015, the well-known AlphaGo developed by Google's DeepMind company utilized the deep learning method to defeat the European Go champion in the Go game. This makes the influence of deep learning increasingly widespread. AI researchers call the current big development of deep learning the third boom of artificial intelligence.

The article "Deep Learning-Based Music Quality Analysis Model" was retracted in 2023. Reasons: signs of a paper mill; suspected computer-generated content; unreliable results or conclusions; lack of ethics approval or compliance.

## 3. Our Proposed Method

Given a music representation, we can analyze it by leveraging a couple of machine learning models, including MLP, CNN, RNN, and their derivatives. For MLP, the input is generally a one-dimensional coefficient vector, such as flattened MFCC. Each learning of MLP is for global features. For CNN, there are many types of acoustic features that can be extracted. When extracting a one-dimensional sound sequence, you can use a 1D CNN for learning and input a two-dimensional spectrogram. Also, you can use a 2D CNN for learning. The main feature of CNN is that it can extract local features and learn the correlation of local features, such as the relationship between adjacent frames, as well as the relationship between adjacent features (frequency dimension). In addition, the weight-sharing network structure of CNN makes its parameters small and the model complexity low. For RNN, we typically model the short-term and long-term correlations (dependencies) at the temporal level. RNN mainly has a good effect on sequence data with strong temporal correlation. For example, the logic before and after speech is a highly informative channel. Usually, CNN and RNN are combined. First, CNN is leveraged to extract high-dimensional features, and subsequently RNN is utilized to characterize temporal correlation. Although RNN performs well on some tasks, there are also other problems. Owing to the long-term dependence of RNN, it is prone to the problem of gradient disappearance. At the same time, it is not as good as CNN on the GPU optimization. Therefore, the training speed is usually a little slow [17]. In addition, GAN also has many applications in music-related signal processing, such as SEGAN for speech enhancement. WaveNet for sound generation and some GAN structures in the field of sound source separation and music instrument conversion are also frequently used.

The high feature descriptiveness of deep learning requires a huge amount of training data. In the domain of music processing, open source datasets are related to speech, such as music-related open source datasets, e.g., Million song Dataset and MusicNet. There are ambient sound-related datasets such as the AudioSet. In addition to the field of speech recognition, other music-related tasks face the problem of small open datasets. We should handle the problem that insufficient data may lead to overfitting of deep networks. Data augmentation can be considered through the idea of random segmentation and random frame skipping, by leveraging the rule-based audio sequence augmentation methods and using random frame skipping. The cyclic neural network is modelled by leveraging multiple predefined rules. The sequence expansion based on the rules is to segment the data and reorganize it sequentially. The random segmentation increases the diversity of the sequence and increases the data size. Also, it can bring significant performance improvement, in order to conduct the shallow learning. The advantages of the deep learning model complement each other, and the decision-making layer fusion method is employed.

The article "Deep Learning-Based Music Quality Analysis Model" was retracted in 2023. Reasons: signs of a paper mill; suspected computer-generated content; unreliable results or conclusions; lack of ethics approval or compliance.

The SVM classifier has a wide range of applications in small-sample music quality evaluation. The PCANET model depends on SVM, which can achieve better results [15]. As a commonly used and effective strategy, SVM adopts the voting mechanism. To summarize, we in this paper propose an effective differential voting mechanism based on voting decision-making. The difference between pairwise SVM classifiers is combined to form the total number of votes, based on which the category with the highest votes is treated as the final decision category. Herein, the SVM classifier using deep learning features is set as D-SVM, and the classifier using shallow learning is the SVM-SVM. We first calculate the difference information of the two models. Afterward, we select a small number of test samples (10 in each category) to test the average recognition ability of the two models. The average music quality recognition rate is *r*_*s*_, and the voting difference information obtained by the two is normalized to the interval [0, 1] according to the quality recognition accuracy. Then, the difference information is distributed: D-SVM is.

(1) $$\begin{array}{c} D_{d}=r_{d}\left(r_{d}+r_{s}\right)*S-D_{d}=r_{d}\left(r_{d}+r_{s}\right), \end{array}$$

wherein *D*_*s*_ = *r*_*s*_ (*r*_*d*_ + *r*_*s*_). Next, we calculate the difference information between each model category. For the “one-to-one” scenario, SVM classifier recognizes *N* categories, given *N*(*N* − 1)/2 sub-classifiers. The classifier votes in pairs according to the distance between each pairwise category. In order to ensure the validity of the votes, invalid votes with a distance less than a prespecified threshold are discarded, which can be described as follows: (1) calculate the threshold *t* (take the average distance value of all sub-classifiers in the sample); (2) abandon the votes with the distance between the two sub-classifiers less than *t*; (3) calculate the final votes of the *N* categories as *V*_1_, *V*_2_, ⋯, *V*_*N*_, where *V*_*i*_ = *D*_*d*_ × *v*_*di*_ + *D*_*s*_ × *v*_*si*_, *v*_*di*_ is the first step of deep learning. The number of valid votes contains*i*categories, and *v*_*si*_ is the number of valid votes for the *i*-th category of shallow learning. Accordingly, the result is max(*V*_1_, *V*_2_, ⋯, *V*_*N*_).

The article "Deep Learning-Based Music Quality Analysis Model" was retracted in 2023. Reasons: signs of a paper mill; suspected computer-generated content; unreliable results or conclusions; lack of ethics approval or compliance.

The music version of Orthoepy attribute evaluation is inseparable from the flag of the auditory example to carefully measure the similarity between the speaker's pronunciation and the color fork. The banner tuning fork is based on the American language when producing music. Meanwhile, the color level is relatively noble, but the evaluation accuracy is not high, which does not hinder the distinction in the characteristics of sonorous color and fashion. In this way, the auditory texture and the experience command cannot be leveraged. Therefore, the auditory patterns are involuntarily slammed to varying degrees to guarantee the accuracy of the music player's assessment of the pronunciation properties. In our work, the regression (MLLR) and maximum posterior probability (MAP) are utilized for other speakers that can disapprove the degree of twinning of auditory dies and touchstone tirade to a certain extent in their own speech [3]]. Moderately overcoming the degree of mismatch is also essential when it is truly useful in the evaluation of English songs ordering, but the degree of authority is still essential after the auditory design is compromised. In GMM-based music recognition, differences are borrowed heavily in the GMM parameters. The MLLR algorithm rule improves on the emergence of narrow innovation-supported adaptive data in estimating sample parameters. Also, the translation normalizing auditory is designed to record experimental conversations and requires only a small amount of data to obtain class events. The MAP algorithm is conducted as estimating the GMM parameters. It can update the Gaussian distribution with attention vector in the adaptive volume. It can also achieve better results in the case of large amount of data. Therefore, in order to fully exploit the advantages of both schemes, the evaluation shape was conditioned by MLLR-MAP model preparation. The Gaussian distribution of HMM fashion uses the same version of the mesh to update all the parameters when the auditory design is set by the MLLR algorithm rule.

It is generally recognized that the MAP algorithm rule is an example of a custom hair split solution. In order to ensure that the flag-level pride can be maintained after the auditory design configuration, the information system automatically recognizes the reading rules. Meanwhile, it eliminates the cuttlefish section with a good face-up as the adaptor. The MLLR-MAP second adaptive auditory dummy [14] is adopted. This technique authorizes American glyphs and digitizes the version words into bold segmentation. It contains the GOP record of metamers. A department that scores more than a preset standard is the inevitability of adapting the subject. This method can achieve a hearing fork that is orthodontic equivalent to a Chinese speaker in English. By thresholding the conspicuous sounds of the phonetic music, we present a face-to-face talk in an age-common analysis. We also position the sign ascent to the English pericope phonetic major. Automated and applied modeling and simulation techniques are suitable for scoring design signature phantoms. Empirical music quality analysis rules are used to quantify and equal utterances. The music eminent is audibly supported by the analysis of the track instance in ripple innovate. The objective of the problem is the citation of the utterance ripple entropy form, wherein the rate fitting of the pronunciation-grade utterances, namely:

(2) $$\begin{array}{c} H_{\text{quality}}=\max\left\{G\left(I^{M},J_{K}\right)-G\left(I^{M},{\text{J}}_{U}^{M}\right)\right\}, \end{array}$$

The article "Deep Learning-Based Music Quality Analysis Model" was retracted in 2023. Reasons: signs of a paper mill; suspected computer-generated content; unreliable results or conclusions; lack of ethics approval or compliance.

## 4. Experimental Results and Analysis

The simulation transport sketch terminates three capabilities: input audio library, network transport model, and distorted audio library. The main factors that affect the streaming media music profession are encoder damage, mesh jitter, and setting damage, so the fret transmission model is embodied in the encoder, packet damage model, and jitter fashion. Among them, the encoder adopts the AMR-WB low berate encoder suitable for streaming media transmission, and the book damage and contractility design are deduced from the recommendations of ITU_T COM12-D97 and ITU-T COM12-D98]. tribune uses 8 encoding methods, 19 shine loss classifications, and 21 levels of jitter. We replace insensitive and undelivered bundles with silent splits when packet loss and irritability occur. According to the requirements of the Chinese harmony classification process in the ITU-T EV-VBR quality evaluation optimization and sorting certification, the atmosphere results are divided into 4 categories: classical orchestra atmosphere, public orchestra, general acapella, and popular acapella_5]. Landing selection 5 vibe results, each with a loop range of 15S, form an input sound bank. For pagan chants and acceptable chants, a disproportionate number of corpora of male and female votes resulted in 2 male languages and 3 female intonations.

20 proof sequences were passed through 48 transmission qualifications, respectively, and 960 permutations were purchased to form a metamorphic descent library. Using the Sphinx4 address recognition system as the carrier, 40 college students were selected to understand English discourse as the main body of the auditory adaptation plan. All students select 20 sentences in the main text and explain in one color voice, even as many as options. The English voice speech database management system mainly includes 70 college students' words. The estimates of bad and socket students are equal, but there are obvious differences in speaking stable. All students declare the meaning of 20 corpora, each with approximately 10 accounts. Three senior English experts were hired as judges to judge the pronunciation characteristics from the aspects of authenticity of eloquence, fluency of eloquence, and integrity of speech. Human scoring is an important foundation of a coach's account and must be Levy first. Taking reactive power reciprocity as the evaluation index, the W scorers are obtained by planting, and the calculated scores are presented in Table 1.

The article "Deep Learning-Based Music Quality Analysis Model" was retracted in 2023. Reasons: signs of a paper mill; suspected computer-generated content; unreliable results or conclusions; lack of ethics approval or compliance.

As can be seen from Table 2, the low degrees of the decision level and the gospel level are 0.84 and 0.79, respectively, indicating that the keyboard has a solid score and can be used as the main messenger of the shape charge. 20% were randomly selected from the address database management system as the test set, and the rest were exercise embarrassment. We calculated the relationship between touchstone events and human graded reasoning and selected an analogy between five-fold break validation to measure and break down machine-graded grades. The acoustic feature extracted from each recorded music. We noticed each recorded feature and identify a broad range of behaviors by attempting a conjoint analysis of SVR scoring patterns. The sources of pronunciation accuracy experience of the music are shown in Table 2. It can be seen from Table 2 that rock obstacle degree and GOP are the best evaluation criteria, and can have good evaluation ability when applied independently, mainly because the GOP score is cream. The correlation between the two can be a good refutation of the authenticity of the pronunciation and can correct the relationship between the clarity of meaning and the directness of the speaker.

In response to the proposition that PEAQ cannot force a moderate evaluation of streaming music , we proposed a PEsAQ metric for music quality evaluation of streaming media. The specific steps are based on imitation. This can be described as follows: (1) Prealign fresh and perverted music first and subsequently remove the quiet music segments before the invention of audio. (2) Design the alignment model and further move the obstacles and irritability of the twisted music through the alignment progress. (3) On the one hand, we use PEAQ to evaluate the configuration of true and distorted music segments and have the evaluation results of PEAQ. On the other hand, the MFCC parameters are descended from the morphing audio and linear morphing music parts, and the DTW fitting of the two is the shortest distance [6]. (4) The objective reason that UDTWoDG conforms to DTW is obtained by analogy, the minimum distance of DTW relation to subjective score. We obtained the DG music as the passport to the operation of obtaining subjective evaluation of the DG music. Alignment model aligns original and malformed music frames as planned. Herein, we performed a skew between perve supported by preserving FFT relation.

The article "Deep Learning-Based Music Quality Analysis Model" was retracted in 2023. Reasons: signs of a paper mill; suspected computer-generated content; unreliable results or conclusions; lack of ethics approval or compliance.

## 5. Conclusions

This paper designed an adaptive evaluation framework for music quality evaluation. Firstly, the music of the vocational evaluation system is proposed. Secondly, the self-adaptive evaluation design of speech characteristics and the verification vector regression algorithm are improved, and the perceptual proofreading is designed based on classification evaluation is demonstrated. Finally, the music quality evaluation standard of the same adaptability is proposed and further empirically evaluated. The rise indicates that the system is able to accurately assess the quality of music recorded from different circumstances. This can show the singer's proficiency and skill. We also noticed that the nonlinear relationship between different acoustic features and autographs ensures the accuracy and consistency of music quality evaluation framework.

## Figures and Tables

**Figure 1:** The flowchart of our proposed music quality evaluation.

**Table 1:** Objective music quality assessment.

Correlation		Music	Player
Different music sections	A	0.642	0.812
	B	0.756	0.784
	C	0.831	0.854
Average score		0.732	0.865

**Table 2:** The fluence of the music players.

Music score		Speed	Duration	Pause	Quality
Correlation level	Sentence	0.54	0.44	0.35	0.84
	Reader	0.67	0.64	0.36	0.79

## Data Availability

The data used to support the findings of this study are available from the corresponding author upon request.
